The article "Role of Iron-Related Oxidative Stress and Mitochondrial Dysfunction in Cardiovascular Diseases" was published in 2022. Journal: Oxid Med Cell Longev.

# Role of Iron-Related Oxidative Stress and Mitochondrial Dysfunction in Cardiovascular Diseases

**DOI:** 10.1155/2022/5124553

**Published:** 2022-09-07

**Authors:** Fang Yan, Kaifeng Li, Wenjuan Xing, Mingqing Dong, Mingliang Yi, Haifeng Zhang

**Affiliations:** ^1^Geriatric Diseases Institute of Chengdu, Department of Geriatrics, Chengdu Fifth People's Hospital, Chengdu, Sichuan Province 611137, China; ^2^Center for Medicine Research and Translation, Chengdu Fifth People's Hospital, Chengdu, Sichuan Province 611137, China; ^3^Teaching Experiment Center Basic Medical Science Academy, Air Force Medical University, Xi'an, Shanxi Province 710032, China; ^4^Department of Aerospace Medicine, Key Laboratory of Aerospace Medicine of the Ministry of Education, Air Force Medical University, Xi'an, Shanxi Province 710032, China; ^5^State Key Laboratory of Space Medicine Fundamentals and Application, China Astronaut Research and Training Center, Beijing 100094, China; ^6^Department of Anesthesiology, Chengdu Fifth People's Hospital, Chengdu, Sichuan Province 611137, China

## Abstract

Iron is indispensable in numerous biologic processes, but abnormal iron regulation and accumulation is related to pathological processes in cardiovascular diseases. However, the underlying mechanisms still need to be further explored. Iron plays a key role in metal-catalyzed oxidative reactions that generate reactive oxygen species (ROS), which can cause oxidative stress. As the center for oxygen and iron utilization, mitochondria are vulnerable to damage from iron-induced oxidative stress and participate in processes involved in iron-related damage in cardiovascular disease, although the mechanism remains unclear. In this review, the pathological roles of iron-related oxidative stress in cardiovascular diseases are summarized, and the potential effects and mechanisms of mitochondrial iron homeostasis and dysfunction in these diseases are especially highlighted.

## 1. Introduction

As an essential micronutrient, iron plays an important role in several biological processes, such as heme synthesis, mitochondrial respiration, DNA synthesis, and iron-dependent catalytic reactions [1]. However, abnormal iron regulation and accumulation has been found to be involved in pathological processes that are associated with many diseases, including cardiovascular diseases, although the underlying mechanisms require further exploration [2, 3]. Excess iron plays key roles in metal-catalyzed oxidative reactions, such as the Fenton reaction, to generate reactive oxygen species (ROS). ROS can cause oxidative stress, lipid peroxidation, aberrant posttranslational modification of proteins, and DNA damage [3].

The article "Role of Iron-Related Oxidative Stress and Mitochondrial Dysfunction in Cardiovascular Diseases" was published in 2022. Journal: Oxid Med Cell Longev.

Mitochondria form the center of oxygen utilization to produce energy, which fundamentally causes the generation of ROS [4]. Furthermore, in mitochondria, iron is used to synthesize heme and to build iron-sulfur clusters in mitochondria; this requires proteins to regulate iron homeostasis that are vulnerable to iron-induced oxidative stress. Aging accompanied by ROS in mitochondria has also been reported to be induced by disruption of iron homeostasis, which is related to mitochondrial decay and dysfunction [5]. However, the relationship between iron-related oxidative stress and mitochondrial dysfunction and their mechanisms in cardiovascular diseases remain unclear.

In this review, iron-related oxidative stress' pathological roles in cardiovascular diseases are summarized, with a focus upon the potential effects and mechanisms of mitochondrial iron homeostasis and dysfunction in these diseases.

## 2. Overview of Iron Homeostasis

### 2.1. Systemic Iron Homeostasis

The amount of iron in adult bodies has been estimated at a total of 3-5 g, where myoglobin and hemoglobin account for two-thirds [3]. The majority of the remaining iron binds to ferritin in the cytoplasm, while extracellular iron accounts for only ~0.1% total body iron [1]. It is the upper jejunum and the duodenum that absorb iron from dietary sources. Gut mucosa cells are able to utilize two distinct mechanisms depending upon whether the iron is in a heme or inorganic form [6]. Iron in the form of heme comprises half of the iron in meat, poultry, and fish. Heme carrier protein 1 (HCP1) is utilized for the absorption of heme in the intestinal epithelial cells' apical membrane [3]. Ferrous iron (Fe^2+^) can be released from heme via degradation by heme oxygenase-1 (HO-1). The absorption of inorganic ferric ion (Fe^3+^) in dietary iron first requires conversion to absorbable Fe^2+^ by cytochrome b reductase 1 (DCYTB) or dietary ascorbate, before being transported across the membrane by divalent metal transporter protein 1 (DMT-1).

Internalized Fe^2+^ enters the cytosolic labile iron pool (LIP) to fulfill cellular needs or is converted to Fe^3+^ for storage via binding to ferritin [1]. Ultimately,1-2 mg/day of dietary iron is usually absorbed, which is usually enough to replace the loss of iron through the blood, skin, urine, and intestinal mucous [7].

Fe^2+^ can be exported through the basolateral membrane by using ferroportin (FPN), after which it is reoxidized to form Fe^3+^ by membrane bound hephaestin. For long-distance delivery via the circulatory system, Fe^3+^ can be bound to transferrin (Tf) [1]. Circulating Tf-bound iron is absorbed by endocytosis into peripheral tissue cells by transferrin receptor 1 (TfR1) [8]. Iron can also be released from the spleen and other organs into the circulation when senescent or damaged erythrocytes undergo macrophage mediated phagocytosis. This iron can be recycled in the bone marrow for heme synthesis [9].

The article "Role of Iron-Related Oxidative Stress and Mitochondrial Dysfunction in Cardiovascular Diseases" was published in 2022. Journal: Oxid Med Cell Longev.

As a peptide hormone, hepcidin is predominately released from the liver. It also plays an important role as a systemic regulator of iron homeostasis [10]. Hepcidin can prevent the efflux of cellular iron through the promotion of FPN internalization and degradation to achieve its effect on systemic iron regulation. Specifically, in enhanced erythropoiesis or iron deficiency conditions (such as hemorrhagic/hemolytic anemia), hepcidin is transcriptionally downregulated causing decreased internalization and degradation of FPN. Thus, macrophages, hepatocytes, and intestinal epithelial cells are more likely to release iron into circulation. On the contrary, when the body is overloaded with iron, e.g., in inflammatory states, hepcidin is overexpressed and promotes FPN internalization and degradation, which prevents cellular iron efflux by the reduction of intestinal iron absorption and iron sequestration in hepatocytes and macrophages. Therefore, the hepcidin-FPN axis is critical for the regulation of systemic iron homeostasis to meet body needs (Figure 1). Further mechanistic understanding of the processes underlying the hepcidin-FPN axis could contribute to the improvement of clinical outcomes for patients with systemic iron imbalance.

### 2.2. Cellular Iron Metabolism

Iron is absorbed into cells in two major ways. Endocytosis is where TfR1 binds to Tf-bound iron to internalize it, whereas DMT-1 is used to transport non-Tf-bound iron (NTBI) into cells [11]. The voltage-gated calcium channels have also been described as transporters of NTBI in cardiomyocytes under iron overload conditions [12]. Iron absorbed by cells enters the redox-active LIP to further be stored in ferritin, assimilated into iron-containing proteins, or utilized by mitochondria to synthesize heme and iron-sulfur (Fe-S) clusters [1, 13].

The posttranscriptional regulation of cellular iron homeostasis is conducted via iron regulatory proteins (IRP1 and IRP2) through interactions with iron-responsive elements (IREs) [14]. IREs are conserved 25-30 nucleotide-long RNA stem-loop structures in the untranslated regions of mRNAs, which encode proteins that participate in iron import (TfR1 and DMT1), export (FPN), and storage (H and L ferritin subunits) [15]. IRPs can stabilize the TfR1 and DMT1 mRNA by binding to IREs located in their 3′Pregion, thereby inhibiting the translation of ferritin and FPN by binding to single 5′IREs [16]. The binding capacity of IRPs to IRE depends upon intracellular iron concentration. The IRE-binding activity of IRPs can be increased when cells are iron deficient with shrunken LIP, TfR1, and DMT-1 mRNA stabilized to enhance iron import and decrease iron export by the suppression of FPN translation. Conversely, IRP-IRE interaction is decreased when cells are iron-repleted with large LIP, resulting in lower TfR1 and DMT1 mRNAs stability and improved ferritin and FPN translation, ultimately enhancing iron storage and release [17] (Figure 1).

The article "Role of Iron-Related Oxidative Stress and Mitochondrial Dysfunction in Cardiovascular Diseases" was published in 2022. Journal: Oxid Med Cell Longev.

Hepcidin is an autocrine protein that has been reported to be produced by the heart for the regulation of iron levels in cardiomyocytes through the hepcidin-FPN1 axis, which can be distinct from systemic iron regulation [18]. For example, cardiac hepcidin is upregulated under hypoxic conditions; whereas systemic hepcidin is downregulated. It is possible that this could be an adaptive mechanism for the maintenance of cardiac function [1, 19].

### 2.3. Mitochondrial Iron Regulation

Iron is important in maintaining mitochondrial function, especially during heme and iron-sulfur (Fe-S) cluster synthesis [20]. Mitochondrial ferritin (FtMt) is a type of ferritin that is particularly expressed in tissues with a high mitochondrial concentration to bind to iron for storage, such as the circulation, central nervous system, testes, thymus, and kidney [21]. Mitoferrin-1 (also known as SLC25A37) with high specificity in hematopoietic tissues was first found in anemic phenotype of Frascati-mutant zebrafish [22]. Mitoferrin-2 (also known as SLC25A28) with widely expression in various tissues was also reported [23]. Mitoferrins located in the inner membrane of mitochondria are thought to be responsible for transporting iron from the cytoplasm into the mitochondria [24]. However, the function of mitoferrins in cardiovascular diseases is still unclear.

ABCB10 is an ATP-binding cassette transporter located within the inner mitochondrial membrane, and it was reported to interact with and stabilize mitoferrin-1 [25]. However, ABCB8 (a different ATP-binding cassette transporter) was found to export iron from the mitochondria [26]. Furthermore, the mitochondrial iron-sulfur cluster exporter ABCB7 also contributes to mitochondrial iron homeostasis [27]. Recent findings indicated that proteins belonging to the NEET family also participate in mitochondrial iron metabolism and homeostasis by transferring cluster/iron to mitochondria [28].

Additionally, iron is used in the mitochondria for synthesizing haem, which aids in catalysis and electron transfer [29]. The production of haem needs eight enzymes, and aminolevulinic acid synthase (ALAS) is responsible for the first rate-limiting stage [30]. The feline leukemia virus subgroup C receptor-related protein 1B (FLVCR1B) transports excess haem in the mitochondria into the cytoplasm and catabolizes it into Fe^2+^, CO, and biliverdin through HO-1 [31]. Furthermore, oxidative stress can induce the production of HO-1 ubiquitously [32]. Haem is exported out of plasma membrane via FLVCR1A [33] and imported into plasma membrane by FLVCR2 [34]. The haem transporter HRG1 and ABCC5 (ATP-binding cassette subfamily C member 5) are two different types of haem transporters, which need further exploration to clarify their functions [35] (Figure 2).

The article "Role of Iron-Related Oxidative Stress and Mitochondrial Dysfunction in Cardiovascular Diseases" was published in 2022. Journal: Oxid Med Cell Longev.

## 3. Iron-Related Oxidative Stress and Mitochondrial Dysfunction

### 3.1. Oxidative Stress Induced by Iron

Reactive oxygen species (ROS) are unstable and reactive molecules that are generated following the utilization of oxygen in the mitochondria and by NADPH oxidase enzymes and cytochromes in cells. Firstly, anion superoxide (O_2_−) is produced for enzymatic conversion to hydrogen peroxide (H_2_O_2_) via superoxide dismutase [36]. H_2_O_2_ has greater stability compared to O_2_− and can cross cellular membranes to act as a signaling molecule provided that their levels remain under a physiologically tolerable threshold, which is controlled by an enzymatically regulated synthesis [37]. However, through the Fenton reaction (requiring transitional metals), H_2_O_2_ is rapidly and efficiently catalyzed to produce hydroxyl radicals (HO), which are the most reactive ROS. As an abundant transitional metal, iron plays key roles in metal-catalyzed oxidative reactions [38].

Iron-catalyzed oxidation mediates lipid peroxidation via reductive cleavage of hydroperoxysides (ROOH) that are obtained from membrane phospholipids, which produce alkoxyl (RO^.^) and peroxyl (RO2^.^) radicals [36]. This formation of lipid radicals is also central to the pathophysiological processes in ferroptosis, where iron-dependent lipid peroxidation drives the process of regulating the death of cells (Figure 3).

### 3.2. Mitochondrial Dysfunction Is Related to Iron-Induced Oxidative Stress

As mitochondria has fundamental roles in creating ROS via oxygen metabolism to produce energy and iron utilization for iron-sulfur cluster assembly and heme synthesis, they tend to be vulnerable to damage from oxidative stress induced by iron.

It was reported that disruption of iron homeostasis in mitochondria can be induced by ROS, which accompanies aging and is related to mitochondrial decay [5]. Mice with heart iron accumulation injected with iron dextran caused mitochondrial DNA damage, which interfered with subunit synthesis in mitochondrial respiration chain, and caused dysfunction of the respiratory system and cardiomyopathy [39]. The accumulation of mitochondrial iron in patients with Friedreich ataxia can be induced by frataxin deficiency (resulting in defective iron sulfur cluster biogenesis), which is accompanied by progressive cardiomyopathy [40, 41].

The article "Role of Iron-Related Oxidative Stress and Mitochondrial Dysfunction in Cardiovascular Diseases" was published in 2022. Journal: Oxid Med Cell Longev.

Mitochondrial iron accumulation and iron-related oxidative stress can also be caused by unregulated iron import and/or export. The absence of ABCB8 (ATP-binding cassette transporter, a mitochondrial iron export protein) can lead to the accumulation of increased mitochondrial iron and oxidative stress, causing cardiomyopathy and increased DOX-induced cardiotoxicity susceptibility [26]. On the contrary, in mitochondria, FtMt prevents oxidative damage caused by iron by modifying the distribution of iron in the cell. A higher expression of FtMt in the heart can protect cardiac mitochondria from DOX-induced oxidative damage [42] .

## 4. Iron-Related Oxidative Stress and Mitochondrial Dysfunction in Ferroptosis

### 4.1. Ferroptosis

In 2012, ferroptosis was reported to be an innovative way of cell death. In contrast to apoptosis, necroptosis, and pyroptosis, ferroptosis has unique genetic, biochemical, morphological, and metabolic characteristics [43]. During ferroptosis, excess intracellular iron accumulation is associated with ROS overproduction, which leads to the extensive oxidation of polyunsaturated fatty acids and damage to the cellular membrane structure, and ultimately cell death [44].

Therefore, iron and iron-related oxidative stress contribute to ferroptosis, since it is an iron-catalyzed accumulation of lethal lipid peroxides that causes the regulation of cell death by iron [45]. Furthermore, when cells undergo ferroptosis, abnormalities of the mitochondria can be detected by electron microscopy. These abnormalities are characterized by the outer membrane rupture, swell, and changes in density. This indicates that mitochondrial dysfunction is associated with ferroptosis [46]. The roles of iron-related oxidative stress and mitochondrial dysfunction in mediating ferroptosis are discussed below.

### 4.2. Iron-Related Oxidative Stress in Ferroptosis

Iron is an important factor that drives ferroptosis, and the accumulation of cellular iron facilitates the Fenton reaction and cytotoxic hydroxyl radicals' production, which subsequently promotes ferroptosis. On the other hand, protective properties against ferroptosis and the Fenton reaction can be derived from a consequence of free ionic iron binding to proteins [47].

Iron uptake via TFR1 can be instrumental for cellular sensitivity to ferroptosis [48], while cytosolic ferritin can control iron availability and confer resistance to ferroptosis [49]. Furthermore, selective ferritin autophagy via NCOA4 can facilitate cellular susceptibility to ferroptosis [50]. The knock down of iron or ferritin exporter expression can promote ferroptosis [51]. The loss of ceruloplasmin promotes the induction of ferroptosis via both erastin and RSL3 (a transcription factor), which helps ferroportin exit cells through its ferroxidase activity [52]. By contrast, poly (rC)-binding protein 1 (PCBP1) knockout mouse hepatocytes have been shown to use this iron chaperone to bind and deliver Fe^2+^ to ferritin. The increased liable iron and lipid peroxidation suggested that PCBP1 can play a role in the prevention of ferroptosis-related disease [53].

The article "Role of Iron-Related Oxidative Stress and Mitochondrial Dysfunction in Cardiovascular Diseases" was published in 2022. Journal: Oxid Med Cell Longev.

### 4.3. Iron-Related Mitochondrial Dysfunction in Ferroptosis

Mitochondrial iron homeostasis is also critical for the prevention of ferroptosis. Mitoferrin-1 and mitoferrin-2 are important mitochondrial iron-import proteins that participate in the biogenesis of heme and Fe-S [23]. Mitoferrin-2 deletion is associated with a reduction of erastin-induced cell death, whereas mitoferrin-2 overexpression can increase ferroptosis [54]. Mitochondrial ferritin can offer protection against ferroptosis, and mitochondria that overexpress ferritin have been shown to be resistant to erastin-induced ferroptosis [55].

The F-S-binding proteins, mitoNEET, and NAF1 participate in mitochondrial iron transportation and have been shown to increase cancer cells' resistance to cell death induced by ROS [55]. Furthermore, increased mitoNEET expression in human hepatocellular carcinoma cells has been shown to prevent ferroptosis induced by erastin [56]. The overexpression of NAF1 in a mouse tumor xenograft model was also demonstrated to confer resistance to sulfasalazine-induced ferroptosis [57]. Suppressing mitochondrial NFS1 (cysteine desulfurase) can sensitize cancer cells to ferroptosis, whereby Fe–S clusters are synthesized using cysteine sulfur [58]. These studies suggest that Fe–S proteins are important for lipid peroxidation during ferroptosis.

The activation of the mitochondrial enzyme, heme oxygenase-1 (HO-1), degrades heme to ferrous iron, which can increase ferroptosis *via* mitochondrial iron overload [59]. Interestingly, a mild increase in the expression of HO-1 could be cytoprotective [60].

## 5. Iron-Related Oxidative Stress and Mitochondrial Dysfunction in Cardiovascular Diseases

### 5.1. Myocardial Ischemia/Reperfusion Injury

Myocardial ischemia/reperfusion (I/R) injury is a common clinical problem following percutaneous coronary intervention (PCI) or thrombolysis for acute myocardial infarction (MI) [61]. The reperfusion of an obstructed coronary artery is required for the restoration of blood flow to enable ischemic zone rescue. However, the I/R-associated excess production of ROS can also cause cardiac damage [62]. Iron overload has been suggested as one of the potential mechanisms underlying myocardial I/R injury. High iron levels have been reported in coronary blood flow in rat hearts subjected to prolonged ischemia, accompanied by increased cardiac cytosolic iron levels [63, 64]. TfR1 expression was increased by hypoxia-inducible factor-1 signaling in myocardial I/R, and upregulation of TfR1 expression was accompanied with increased iron content in I/R-treated rat hearts, which may be the cause for iron overload in I/R [65, 66].

The article "Role of Iron-Related Oxidative Stress and Mitochondrial Dysfunction in Cardiovascular Diseases" was published in 2022. Journal: Oxid Med Cell Longev.

As mitochondria are central to metabolic stresses as essential sources of ROS, mitochondrial dysfunction being caused by oxidative stress can lead to cell death during I/R injury [67]. The increase in iron deposition, ROS production, and cardiomyocyte apoptosis was reported in hereditary hemochromatosis (HFE) mice after I/R injury [68]. Furthermore, increased mitochondrial iron was detected following myocardial I/R injury in mice and ischemic cardiomyopathy in human cardiac specimens. It is notable that *in vivo* protection against I/R damage was achieved via the pharmacological reduction of mitochondrial iron [69].

FOXC1-mediated transcriptional activation of ELAVL1 was reported to increase myocardial I/R-associated ferroptosis via autophagy modulation and cause myocardial injury [70]. MiR-135b-3p also promoted myocardial I/R injury by reducing GPX4 expression [71]. The long noncoding RNAs (lncRNAs) LncAABR07025387.1 was also found to upregulate acyl-CoA synthetase long-chain family member 4 (ACSL4)-mediated ferroptosis and finally enhanced myocardial I/R injury [72].

It has been reported that ferroptosis occurs in diabetic myocardial I/R injury with endoplasmic reticulum stress [73]. The inhibition of DNMT-1 during diabetes-associated myocardial I/R injury was shown to alleviate ferroptosis via NCOA4-mediated ferritinophagy [74], whereas Naringenin (a flavonoid) was reported to reduce ferroptosis and myocardial I/R injury through a nuclear factor-erythroid factor 2-related factor 2 (Nrf2)/System xc^−^/GPX4 regulatory axis [75]. Baicalin, a natural flavonoid glycoside, can also impede myocardial I/R injury by inhibiting ACSL4-mediated ferroptosis [76]. Likewise, etomidate has been shown to attenuate ferroptosis via the Nrf2/HO-1 pathway in a rodent model of myocardial I/R [77].

### 5.2. Atherosclerosis

In patients with atherosclerotic lesions, iron deposition was reported to be associated with increased cholesterol levels [78]. It was also found that plaques were more likely to have higher concentrations of iron and a higher risk of cap rupture in symptomatic patients when compared with plaques from asymptomatic patients [79]. The notion that iron may stimulate the development of atherogenesis has been widely investigated.

The article "Role of Iron-Related Oxidative Stress and Mitochondrial Dysfunction in Cardiovascular Diseases" was published in 2022. Journal: Oxid Med Cell Longev.

Endothelial cells, monocytes/macrophages, vascular smooth muscle cells, and platelets that experience iron overload have all been shown to participate in atherosclerosis. Iron's pathological involvement in atherogenesis may depend upon a catalytically active form for generating ROS and inducing lipid peroxidation within cells that form atherosclerotic lesions [1, 80]. Excess iron also appears to have an atherogenic role in the promotion of macrophage differentiation to produce foam cells via the modification of low-density lipoproteins [1]. Iron overload was reported to drive endothelial cell dysfunction due to its prooxidant/inflammatory effects and promote the phenotypic switch in smooth muscle cells of the vascular system, which was also associated with increased proliferation, ROS production, and apoptosis [81]. It was also found that iron overload can enhance macrophage glycolysis and inflammation and exacerbate the development of atherosclerosis [82].

Ferroptosis has been observed during atherosclerosis initiation and development, whereas inhibition of ferroptosis in murine aortic endothelial cells has been shown to alleviate atherosclerosis via the attenuation of lipid peroxidation and endothelial dysfunction [83]. Prenyl diphosphate synthase subunits 2 (PDSS2) was reported to play a cardioprotective role by inhibiting ferroptosis by activating Nrf2 in atherosclerotic vascular endothelial cells [84]. In diabetic atherosclerosis, HMOX1 (heme oxygenase) knockdown in human endothelial cells attenuated Fe^2+^ overload, which reduced ROS levels and alleviated lipid peroxidation and reduced ferroptosis [85].

microRNA-132 (miR-132) was determined to promote atherosclerosis by inducing mitochondrial oxidative stress-mediated ferroptosis [86]. High level of uric acid (HUA)-induced ferroptosis in macrophages was associated with atherosclerotic plaque formation, which promoted atherosclerosis by targeting NRF2 [87]. Therefore, iron-related oxidative stress and ferroptosis can help enhance the understanding of atherosclerotic pathological processes and perhaps provide novel therapeutic targets.

### 5.3. Doxorubicin (DOX)-Induced Cardiomyopathy

Doxorubicin (DOX) is a member of the antitumor anthracycline family, which comprise some of the chemotherapeutic drugs that are most effective for many malignancies. However, DOX usage is limited in the clinic due to the potential for cardiomyopathy and the development of congestive heart failure [15]. Iron's role in cardiotoxicity induced by DOX has been determined by many studies. For example, mice lacking HFE had increased DOX-dependent cardiac damage susceptibility; this model is particularly interesting since it mimics the iron overload associated with hereditary hemochromatosis in humans [88]. However, the molecular mechanisms underlying the process by which iron overload promotes the exacerbation of these cardiotoxic effects are not yet fully understood.

The article "Role of Iron-Related Oxidative Stress and Mitochondrial Dysfunction in Cardiovascular Diseases" was published in 2022. Journal: Oxid Med Cell Longev.

It was found that ferroptosis inhibition significantly enhanced cardiac function and reduced mortality in a DOX-induced cardiomyopathy mouse model, which proved to be related to free cellular iron release via the upregulation of HO-1 [89]. Furthermore, DOX treatment induced ferroptosis, which was predominantly triggered in the mitochondria by downregulating GPX4 [1]. Acyl-CoA thioesterase 1 (a key fatty acid metabolism enzyme) was found to exert an antiferroptosis effect in DOX-mediated cardiotoxicity [90].

Protein arginine methyltransferase 4 (PRMT4) participates in the regulation of transcription, particularly oxidative stress and autophagy modulation, and can promote ferroptosis during DOX-induced cardiomyopathy by inhibiting Nrf2/GPX4 signaling [91]. Fisetin, an abundant flavonoid in fruits and vegetables, attenuated DOX-induced cardiomyopathy via the inhibition of ferroptosis by activating SIRT1/Nrf2 signaling [92]. Salidroside was also demonstrated to have a cardioprotective role in DOX-induced cardiomyopathy by significantly reducing ferroptotic cell death via AMPK-dependent signaling pathway activation [93]. The protective effect of dexrazoxane in the reduction of cytotoxicity in DOX-induced cardiomyopathy in rats was proven to inhibit ferroptosis by regulating high mobility group box 1 (HMGB1) [94]. These studies highlight that iron-related oxidative and ferroptosis have an important role in DOX-induced cardiomyopathy and could provide potential therapeutic targets.

### 5.4. Diabetic Cardiomyopathy

Left ventricular dysfunction, cardiac fibrosis, myocardial hypertrophy, and intracellular accumulation of lipid peroxide are characteristic features of diabetic cardiomyopathy (DCM), which is the predominant factor affecting diabetic patients' morbidity and mortality [95]. It was reported that inhibition of the ZFAS1 reduces ferroptosis by acting as a sponge for miR-150-5p and leads to the activation of CCND2 against DCM in cardiomyocytes following high glucose exposure and in left ventricular myocardial tissues from db/db mice [96]. The inhibition of cardiac autophagy can also activate Nrf2-mediated ferroptosis, which can lead to myocardial damage in murine models of type 1 diabetes [97]. Ferroptosis was further reported to be essential for DCM, where Nrf2 is activated following the sulforaphane-mediated inhibition of cardiac cell ferroptosis due to the upregulation of ferritin and SLC7A11 levels [98].

The article "Role of Iron-Related Oxidative Stress and Mitochondrial Dysfunction in Cardiovascular Diseases" was published in 2022. Journal: Oxid Med Cell Longev.

There is a need for further research to explore the effects and underlying mechanisms associated with iron-related oxidative stress and mitochondrial dysfunction in the development of DCM.

### 5.5. Hypertension

The prevalence of hypertension was positively correlated with serum ferritin by two studies conducted in Korea [99]. The risk of high blood pressure and incidence of hypertension were also found to be positively correlated with hemoglobin and transferrin levels according to a large longitudinal study in China [100]. The sympathetic overactivation detected in patients with hypertension and iron overload was related to elevated serum ferritin, which possibly participated in the increased cardiovascular risk.

Interestingly, cardiac risk was increased in patients with hypertension and iron overload because of elevated serum ferritin levels [101]. Dahl salt-sensitive rats with hypertension were attenuated from hypertrophy, fibrosis, and inflammation of the cardiovascular system when dietary iron was restricted [102]. Additionally, restricting dietary iron prevented the progress of hypertension and kidney fibrosis in a murine model of aldosterone/salt-induced hypertension [103].

*Eucommia ulmoides Oliver*- L. has recently been reported to regulate ferroptosis through the neurovascular-related ligand-receptor interaction pathway and considered to have the potential of treating hypertension and preventing ischemic stroke [104].

This data suggests that the dysregulation of iron metabolism may contribute to hypertension independently. Ferroptosis and components from natural products for its prevention represent new fields that are exploring iron-related oxidative stress in systemic hypertension.

## 6. Therapeutic Potential of Targeting Iron-Related Oxidative Stress and Mitochondrial Dysfunction in Cardiovascular Diseases

Iron depletion by using iron chelators is considered to be a potential treatment for cardiovascular diseases due to the important role that iron-related oxidative stress and mitochondrial dysfunction play in their development. Iron chelation has been observed as improving contractile function in some animal models by increasing cell viability, attenuating cardiac remodeling, and reducing infarction size after I/R injury [89]. However, this relationship was not reproducible in some other *in vivo* models. It was also reported that a cell-permeable iron chelator, 2,2′-bipyridyl, protected the heart from I/R injury, but desferrioxamine (DFO) which has low cellular permeability did not have the same protective effects [69]. The clinical application of this therapeutic strategy requires further studies.

The article "Role of Iron-Related Oxidative Stress and Mitochondrial Dysfunction in Cardiovascular Diseases" was published in 2022. Journal: Oxid Med Cell Longev.

Ferroptosis has also been reported in cardiomyocyte damage induced by I/R. Indeed, the targeting of ferroptosis may prove to be valuable for patients with a diverse array of I/R conditions [89]. I/R-associated heart injury can also be attenuated by blocking ferroptosis via the inhibition of glutaminolysis [48]. A protective effect was observed via the inhibition of USP19/Beclin1-mediated ferroptosis with Cyanidin-3-glucosides in a rat model of myocardial I/R injury [105]. Mitochondria-specific GPX4 overexpression contributes significantly to preventing lipid peroxidation, alleviating cardiac dysfunction following I/R by attenuating ferroptosis [106]. Thus, the targeting of ferroptosis may be able to provide potential prevention strategies for myocardial injury caused by I/R.

As iron deposition and lipid oxidative modification are observed in plaques during atherosclerotic development, ferroptosis is considered to participate in the process. DFO-based iron chelation therapy has inhibited the development of atherosclerotic lesions, which suggests the potential therapy to prevent atherosclerosis by targeting ferroptosis [107]. In DOX-treated murine hearts, it was reported that acyl-CoA thioesterase 1 might have an antiferroptosis impact in cardiotoxicity induced by DOX [90]. The findings of these studies indicate that ferroptosis might also be a potential therapeutic target to prevent DOX-induced cardiomyopathy.

The mitochondria have their own set of proteins to regulate iron homeostasis. FtMt is only present in mitochondria and possesses ferroxidase activity and is essential in acute exhaustive exercise-induced myocardial injury via the modulation of cellular survival and ROS regulation [108]. These findings suggest that regulation of mitochondrial iron can provide potential therapeutic targets to treat myocardial injury due to its unique cohort of proteins. These targets may prove to be especially effective due to the essential role of mitochondria in I/R injury.

## 7. Conclusions and Future Directions

The mineral iron is essential to maintaining normal physiological processes. However, iron-related oxidative stress and mitochondrial dysfunction can also participate in the pathological development of cardiovascular disease, especially I/R, atherosclerosis, DOX induced cardiomyopathy DCM, and hypertension (Figure 4). Ferroptosis regulates cell death through the signaling of lipid peroxidation mediated by iron, and it is an important mechanism responsible for iron-related oxidative stress and mitochondrial dysfunction. The therapy of iron chelation has been proven to be efficacious for the prevention of cardiovascular diseases in many studies. This therapy may target iron-related oxidative stress and mitochondrial dysfunction and ferroptosis. However, future studies are necessary to determine its safety and efficacy with more attention to specific cardiovascular diseases and the peculiarity of iron chelators. Moreover, the critical role of mitochondrial iron homeostasis and dysfunction is slowly being understood in the processes involved with iron-related oxidative stress and the acceleration of cardiovascular disease pathology. The specific targeting of mitochondrial iron regulation and iron-related oxidative stress in mitochondria may provide potential therapies for the treatment of cardiovascular diseases.

The article "Role of Iron-Related Oxidative Stress and Mitochondrial Dysfunction in Cardiovascular Diseases" was published in 2022. Journal: Oxid Med Cell Longev.

## Figures and Tables

**Figure 1:** Systemic iron homeostasis and cellular iron metabolism [1]. In the gut mucosa, Fe^3+^ is converted to Fe^2+^ by DCYTB and then transported by DMT1, whereas haem is transported by HCP1. Intracellularly, Fe^2+^ is released from haem by heme oxygenase-1 (HO-1). Fe^2+^ is converted to Fe^3+^ and bound by ferritin for storage or released via ferroportin (FPN) and converted to Fe^3+^ by hephaestin. Fe^3+^ is transported by binding to transferrin in circulation and is taken up by transferrin receptor-mediated endocytosis into cells for storage (ferritin), release (FPN), and utilization of mitochondria. Iron regulatory proteins (IRP1 and IRP2) regulate cellular iron homeostasis through interactions with iron-responsive elements (IREs), to enhance iron uptake by stabilizing the mRNA of transferrin receptor and DMT-1 and inhibit iron excretion by suppressing FPN translation. Hepcidin can bind to FPN and inhibit its function in iron absorption and iron mobilization from stored pools. Abbreviations: DCYTB: cytochrome b reductase 1; DMT-1: divalent metal transporter protein 1; FPN: ferroportin; HCP1: heme carrier protein 1; HO-1: heme oxygenase-1; IREs: iron-responsive elements; IRP: iron regulatory proteins; LIP: labile iron pool.

**Figure 2:** Mitochondrial iron regulation [109]. The transport of iron across the mitochondrial membrane is mediated by mitoferrin-1 with assistance from ABCB10 and mitoferrin-2. Iron in the mitochondria is mainly used to synthesize iron–sulfur (Fe-S) clusters by NFS1 (cysteine desulfurase) and haem by ALAS (aminolevulinic acid synthase), while excess iron can be stored in mitochondrial ferritin (FtMt). The export of Fe-S clusters into the cytoplasm might require iron–sulfur cluster transporters ABCB7, ABCB8, NAF-1, and mitoNEET, whereas haem efflux into the cytoplasm is promoted by FLVCR1B (feline leukemia virus subgroup C receptor-related protein 1B). Abbreviations: ABCB: ATP-binding cassette transporter; Ala: 5-aminolevulinate; CO: carbon monoxide; Cys: cysteine; ETC: electron transport chain; FLVCR: feline leukemia virus subgroup C receptor-related protein; FtMt: mitochondrial ferritin; HO-1: heme oxygenase-1; NAF1: nuclear assembly factor 1; NFS1: cysteine desulfurase; OXPHOS: oxidative phosphorylation; DADH: reduced form of nicotinamide-adenine dinucleotide; TCA: tricarboxylic acid.

The article "Role of Iron-Related Oxidative Stress and Mitochondrial Dysfunction in Cardiovascular Diseases" was published in 2022. Journal: Oxid Med Cell Longev.

**Figure 3:** Iron-related ROS generation and oxidative stress [4]. Anion superoxide (O_2_∙^−^) is produced following oxygen utilization by oxidative phosphorylation (OXPHOS) and is converted to hydrogen peroxide (H_2_O_2_) by superoxide dismutase enzyme (SOD). H_2_O_2_ is rapidly and efficiently catalyzed by Fe^2+^ through the Fenton reaction to originate hydroxyl radicals (HO∙), the most reactive ROS. Fe^2+^ and Fe^3+^ also mediate membrane lipid peroxidation by catalyzing the reductive cleavage of hydroperoxysides (ROOH) resulting in the production of alkoxyl (RO∙) and peroxyl (RO2∙) radicals. Abbreviations: H_2_O_2_: hydrogen peroxide; HO∙: hydroxyl radicals; O_2_∙−: anion superoxide; OXPHOS: oxidative phosphorylation; ROOH: hydroperoxysides; RO∙: alkoxyl; RO2∙: peroxyl; ROS: reactive oxygen species; SOD: superoxide dismutase.

**Figure 4:** A schematic summary of iron-related oxidative stress and mitochondrial dysfunction in cardiovascular diseases. Abbreviations: ACSL4: acyl-CoA synthetase long-chain family member 4; ACOTs: acyl-COA thioesterases; ADRB2: adrenoceptor beta 2; AMPK: adenosine monophosphate-activated protein kinase; CCND2: cyclin D2; CHRM1: cholinergic receptorM1; DNMT-1: DNA (cytosine-5)-methyltransferase 1; ELAVL1: embryonic lethal-abnormal vision like protein 1; FOXC1: forkhead box C1; FTH1: ferritin heavy chain-1; GPX4: glutathione peroxidase 4; HIF-1: hypoxia-inducible factor 1; HMGB1: high mobility group box 1; HMOX1: heme oxygenase-1; HO-1: heme oxygenase-1; HUA: high levels of uric acid; NCOA4: nuclear receptor coactivator 4; Nrf2: erythroid factor 2-related factor 2; NR3C1: nuclear receptor subfamily 3 group C member 1; OPRD1: opioid receptor protein; PCBP2: poly (C)-binding protein 2; PDSS2: prenyl diphosphate synthase subunit 2; PRMT4: protein arginine methyltransferase 4; ROS: reactive oxygen species; SIRT1: NAD-dependent protein deacetylase sirtuin-1; SLC3A2: solute carrier family 3 member 2; SLC7A11: solute carrier family 7 member 11; TfR1: transferrin receptor 1; ZFAS1: zinc finger antisense 1.

The article "Role of Iron-Related Oxidative Stress and Mitochondrial Dysfunction in Cardiovascular Diseases" was published in 2022. Journal: Oxid Med Cell Longev.

## Data Availability

The data used to support the finds of this study are available from the corresponding author upon request.
